This article has been retracted.

# Safety and Efficacy of Unicondylar Knee Prosthesis Treatment for Unicompartmental Osteoarthritis of the Knee Joint

**DOI:** 10.1155/2022/2938380

**Published:** 2022-07-15

**Authors:** Dahua Zhang, Xiang Zhang

**Affiliations:** Department of Orthopedics, The First Affiliated Hospital of Xi'an Medical University, 710000, China

## Abstract

**Background:**

Knee osteoarthritis (KOA) is a chronic disease that seriously endangers the health of the elderly. Choosing appropriate surgery for knee osteoarthritis patients is especially important.

**Objective:**

To investigate the safety and efficacy of unicondylar knee prosthesis treatment for unicompartmental osteoarthritis of the knee.

**Materials and Methods:**

One hundred patients with unicondylar osteoarthritis of the knee treated in our hospital from June 2019 to June 2021 were selected as retrospective study subjects and were divided into 50 cases each in the comparison group and the observation group according to the different surgical methods. Among them, the comparison group was treated with unicondylar knee arthroplasty (UKA), and the observation group was treated with unicondylar knee prosthesis replacement, and the differences in AKS score, knee flexion angle, tibial angle orthosis, joint mobility, and postoperative recovery were compared between the two groups.

**Results:**

The AKS score and knee flexion angle score of the observation group were higher than those of the comparison group after surgery. However, the tibial angle orthopedic score of the observation group was significantly lower than that of the comparison group after surgery for comparison, and the VAS score of the observation group was lower than that of the comparison group. However, the Lysholm score of the observation group was higher than that of the control group after surgery (*P* < 0.05). The complication rate of patients in the observation group was significantly lower than that of the comparison group, and the HSS score, VAS score, and knee mobility (ROM) of the two groups were statistically significant (*P* < 0.05) when compared at 7 d after surgery and 6 months after surgery.

**Conclusion:**

The clinical efficacy of unicondylar knee prosthesis replacement for osteoarthritis of the knee is better than that of unicondylar knee arthroplasty (UKA) treatment.

## 1. Introduction

In the physiological structure of the human body, the knee joint is one of the most important joints in motion. Its anatomical structure is complex, and it is susceptible to functional damage caused by external forces and other factors, which seriously affects the quality of life and daily activities of patients [1]. Unicompartmental knee osteoarthritis is a chronic degenerative disease characterized by degeneration and loss of articular cartilage and osteophytes of the articular margins and subchondral bone, mostly occurring in middle-aged and elderly people. Lesions can involve unicompartmental and multicompartment, unicompartmental lesions are the predominant in the early stage, and the medial compartment is more common [2].

Gunston [3] invented a prosthesis that could limit knee motion, and one of the other major inventions was that it used a mixture of materials to form a prosthesis. Marmor [4] designed the first unrestricted unicondylar joint prosthesis based on previous generations of unicondylar prostheses, which improved the patient's function. Marmor summed up the clinical experience of previous failures and found that the subsidence of the peritibial component may be related to the width of the tibial part of the component not being wide enough to support the tissue, so the size of the tibial component was increased to ensure greater support around the tibia to prevent the tibial prosthesis sinks. Unicompartmental knee arthroplasty (UKA) is currently the most commonly used surgical method of treating KOA in clinical practice and has also been widely used in knee monoventricular osteoarthritis in recent years. During this period, further development of the UKA was limited for a variety of reasons, the more common of which was the tendency of the peritibial prosthesis to sink, leading to early prosthetic loosening. After the great development of total knee replacement, Scott et al. [5] designed a unicondylar prosthesis (Oxford unicondylar prosthesis) that simulated normal knee motion, based on the success of the artificial total knee. The spacer of the Oxford unicondylar prosthesis is movable, which well reduces the problem of poor mobility of the restrictive prosthesis. Still, the clinical trial found that this unicondylar prosthesis often leads to dislocation of the prosthesis due to the high mobility. With the further development of prosthetic materials and devices, unicondylar replacement surgery has also progressed more significantly [6, 7].

Knee arthroplasty is a safe and effective treatment method for knee joint injuries using artificial knee prostheses for replacement and replacement in recent years [8]. With the continuous progress of science and technology, knee prosthesis design has gradually become one of the key topics that cannot be ignored in knee arthroplasty. Currently, knee arthroplasty is widely used in developed countries. However, caution is still required for the selection of artificial knee replacement, as the replacement prosthesis cannot be replaced at will, and replacement is costly. Hence, the selection of an appropriate artificial knee prosthesis becomes a key issue in replacement surgery.

## 2. Material and Methods

### 2.1. Research Object

One hundred patients with unicompartmental knee osteoarthritis treated in our hospital from June 2019 to June 2021 were selected for the retrospective study and were divided into 50 cases each in the comparison group and observation group according to the surgical modality. These patients were operated on only one side of the knee later, and all cases were free of serious cardiopulmonary and other important organ dysfunctional diseases, and all controlled their blood glucose and blood pressure within the ideal range and had good mental status during the perioperative period. The following are the indications for unicondylar replacement [9]: age ≥ 60 years, body mass < 82 kg, relatively low activity, morning stiffness of the knee < 30 min, persistent pain, knee mobility ≥ 90°, flexion contracture < 5°, inversion deformity ≤ 10°, or valgus deformity ≤ 15°. There were no patients who could not cooperate with the study, and there were no absent or withdrawn patients.

### 2.2. Diagnostic Criteria

The diagnostic criteria for unicompartmental osteoarthritis of the knee followed the criteria for unicompartmental osteoarthritis of the knee in the Osteoarthritis Treatment Guidelines (2018 edition) [10]. The preoperative diagnosis was consistent with knee osteoarthritis, complaints of anterior medial knee pain, or mild patellofemoral joint pressure pain, no lateral patellofemoral joint pain, limited pressure points in the medial joint space, negative physical examination drawer test and lateral stress test, and no flexion deformity, and preoperative X-ray showed that the patient had medial compartment osteoarthritis and the patellofemoral joint was not involved or was only mildly involved.

### 2.3. Inclusion and Exclusion Criteria

Inclusion criteria are as follows: (1) obesity, youth and high activity level, joint disease rheumatoid arthritis, villous nodular synovitis), contralateral interval and patellofemoral degeneration, and anterior cruciate ligament injury; (2) only unilateral interval space narrowing or loss in the weight-bearing phase of the knee X-ray, no cartilage softening, or only mild degeneration in the other intervals; (3) patients with structurally intact joint ligaments, noninflammatory arthritis, low postoperative activity, and low functional requirements; (4) all patients gave informed consent to this study and signed the informed consent form voluntarily; and (5) proposed surgical treatment in line with the indications for surgery.

Exclusion criteria are as follows: (1) with significant resting pain, the presence of moderate or more softening of the patellofemoral joint, and exposed sclerotic subchondral bone; (2) the lateral compartment with severe damage to the meniscus and anterior cruciate ligament, with diseases such as gout or rheumatoid arthritis; (3) the degree of knee flexion contracture, those who are still greater than 15° after passive correction, medial collateral ligament instability, or those who show laxity of more than 2 mm, HT0 surgery, and those who are more active and weigh more than 100 kg; (4) history of previous knee trauma and surgery on the affected side; (5) patients with major organ dysfunction; (6) diseases of the hematologic system and immune dysfunction; (7) unable to cooperate with the research, lost to follow-up or withdrew; and (8) concomitant mental illness.

## 3. Methods

### 3.1. UKA Treatment

In the comparison group, the patient was treated with unicondylar knee arthroplasty (UKA). After anesthesia, the patient was placed in a supine position, a tourniquet was applied to the affected limb and routine disinfection was performed, and a sterile surgical sheet was laid. The anterior medial incision of the left knee was made about 10 cm, and the skin, subcutaneous tissue, and deep fascia were incised, and the knee joint was incised on the medial side of the patella up to 1 cm below the patellar ligament stop of the tibial tuberosity, and the joint fluid was aspirated. After adequate release of the soft tissue, the lesion was viewed to confirm that the osteoarthritis was confined to the medial compartment, with no accumulation in the lateral compartment, and to probe the integrity of the ACL. The medial tibial bone tissue was intercepted with a tibial locator rod placed in the appropriate position. The femoral positioning rod is inserted to determine the osteotomy position of the medial femoral condyle, and an appropriate amount of bone tissue is removed. Insert the tibial plateau prosthesis into the trial mold, and flex and extend the knee joint to show moderate soft tissue tension with equal clearance. Decide on the appropriate type of prosthesis. The bone surface is flushed with pulses, the bone cement is prepared, the tibial and femoral prostheses are fixed in sequence, tapped, excess bone cement is removed, and pressure is applied until the bone cement cures. The peripatellar rim was trimmed and denervated by electrocautery. A polymer polyethylene liner was placed and the knee was flexed and extended, showing knee mobility (flexion) of 130°-0° (extension) with good patellar trajectory and moderate internal and external tension. The Oxford 3 generation unicondylar device used in our hospital was counted for gauze and instruments without error, one drain was left in place, and the incision was closed layer by layer. An elastic bandage was wrapped, a tourniquet was loosened, and the drainage tube was attached to the drainage device.

### 3.2. Unicondylar Knee Prosthesis Replacement

The observation group was treated with unicondylar knee prosthesis replacement, and all patients were routinely infused with cefazolin pentahydrate 1.0 g intravenously 30 minutes before surgery to prevent infection. In the supine position, a tourniquet was placed on the root of the affected thigh on top of a brace, and the knee joint was fully extended until it reached at least 120° of flexion. After satisfactory anesthesia, the knee is flexed 90 degrees, and a parapatellar incision is made from 0.5 cm from the superior medial edge of the patella, obliquely down to the medial tibial tuberosity, with a length of about 8 cm, to fully expose the surgical area and perform an L-shaped incision of the joint capsule, pushing only the patella laterally, without externalizing the patella. The three compartments of the knee joint and the anterior and posterior cruciate ligaments are explored to confirm whether a change in the surgical approach is required. Subsequent resection of the femur, tibia and patella at the bony tubercle and medial meniscus A tibial guide is fitted and the osteotomy is maintained at about 5-7° posterior tilt. Measure the cut tibial plateau with a grinder to determine the plateau size. Install the femoral drilling guide to ensure accurate alignment and then perform femoral drilling. After completing the femoral osteotomy, the femoral condyle is ground and excess tissue is removed. The tibial and femoral prostheses (Oxford third generation unicondylar prosthesis) were selected according to the actual situation and fixed with bone cement. The joint movement was checked, the wound was fully irrigated, a cocktail of saline, ropivacaine 180 mg, epinephrine 0.2 mg, and morphine 10 mg were injected into the joint capsule, a drainage tube was placed, the joint capsule was tightly sutured, and the subcutaneous and skin were sutured in turn and wrapped with an adjuvant. To prevent the formation of deep vein thrombosis (DVT) in both lower extremities after surgery, patients were instructed to take oral rivaroxaban 10 mg anticoagulation 6 hours after surgery and then one tablet daily until 35 days after surgery. The hematocrit should be transfused if it was lower than 70 g/l, and those with 70 g/l-90 g/l should be treated according to their actual physical condition.

In both groups, the drainage tube was removed within 24 h after surgery, and knee flexion and extension exercises were performed after the removal of the tube, and the use of a walker or crutches was encouraged. Cefazolin pentahydrate 1.0 g twice daily was used routinely for 3 days after surgery to prevent infection. Parecoxib 100 ml was used every twelve hours for pain relief (40 mg+0.9% sodium chloride injection 100 ml) for 3 days after surgery and then changed to celecoxib 200 g twice daily orally after 3 days. Individual patients were treated symptomatically. Both groups of patients had their incisions removed on the 14th postoperative day, and front and side X-rays of both knees were taken on the second postoperative day to observe the position of the prosthesis.

### 3.3. Observation Indicator

(i) The American Knee Score (AKS) was used to assess the knee function before and after surgery in both groups. The total score was 100, and the higher the score, the better the recovery of the knee function. (ii) The VAS and Lysholm scores were compared before and after surgery in both groups, with a total score of 100 points, based on the total assessment score to determine the patient's joint function, poor: <60 points, moderate: 60-70 points, good: 7180 points, and excellent: ≥81 points. (iii) Knee US Hospital for Special Surgery (HSS): with a total score of 100 points, based on the higher the total assessment score, the better the patient's joint function situation. Postoperative pain was assessed by VAS, which was assessed as less than 3 points for mild pain, 4~6 points for pain and interfering with sleep, and 7~10 points for intense pain in both groups, comparing the pain level before and after the intervention in both groups.

### 3.4. Statistical Analysis

All statistical data in this study were entered into excel software by the first author and the corresponding author, respectively, and the statistical processing software was SPSS25.0 for calculation. Repeated measures analysis of variance between groups was used to measure the measurement expressed as mean ± standard deviation (*X* ± SD). *χ*^2^ tested count data expressed as a percentage (%). Univariate and logistic multivariate regression analysis was used to compare the influencing factors, and the risk factors with significant differences were screened. Correlation test using logistic regression linear correlation analysis was used. Included data that did not conform to a normal distribution was described by M(QR), using the Mann-Whitney test. All statistical tests were two-sided probability tests. The statistical significance was *P* < 0.05.

## 4. Results

### 4.1. General Data Analysis

There was no significant difference between the two groups regarding gender, average age, body mass index, Ahlback classification, and other general data by *t*-test and chi-square test (*P* > 0.05). See Table 1.

### 4.2. AKS Score, Knee Flexion Angle, and Tibial Angle Correction

Before surgery, the differences in AKS score, knee flexion angle, and tibial angle orthosis between the two groups were not statistically significant (*P* > 0.05). After surgery, the AKS score and knee flexion angle of the observation group were higher than those of the comparison group. However, the tibial angle orthosis of the observation group was significantly lower than that of the comparison group after surgery, and this difference was statistically significant (*P* < 0.05). See Figure 1.

### 4.3. Comparison of Joint Mobility

Before surgery, there was no statistically significant difference between the VAS and Lysholm scores of the two groups (*P* > 0.05); after surgery, the VAS score of the observation group was lower than that of the comparison group. However, the Lysholm score of the observation group was higher than that of the control group after surgery, and the difference was statistically significant (*P* < 0.05). See Figure 2.

### 4.4. Comparison of Postoperative Recovery

There was a statistically significant comparison of HSS scores and knee mobility (ROM) between the two groups at 7 d and 6 months postoperatively (*P* < 0.05). There was no statistically significant comparison of HSS scores and ROM between the two groups at the final follow-up (*P* > 0.05). See Figure 3.

### 4.5. Complication Comparison

Comparing the complications between the two groups, the incidence of complications in the observation group was significantly lower than that in the control group, and the difference was statistically significant (*P* < 0.05). See Figure 4.

## 5. Discussion

Unicondylar knee replacement is used to replace the damaged cartilage surface of the tibiofemoral joint of the knee, which is only suitable for early unicondylar osteoarthritis of the knee. It has the advantages of less trauma, quick recovery, less complications, and high patient acceptance [11]. However, its scope of surgical indications is narrower than that of total knee replacement due to its high patient selection requirements; at the same time, the technique of total knee replacement is more mature and its efficacy is far from certain [12]. Unicondylar knee replacement is currently used in a small range, which long-term clinical efficacy still needs further clinical verification [13]. However, if the indications for surgery are accurately grasped, appropriate patients are selected, and careful preoperative preparations and skilled surgical operations are performed, the clinical results are satisfactory [14, 15]. The advancement of surgical techniques unicondylar replacement of the knee applied to anteromedial compartment osteoarthritis of the knee has a broad prospect with the improvement of prosthesis and instrumentation design.

In our study, the AKS score and knee flexion angle score of the observation group after surgery were higher than those of the comparison group. However, the tibial angle orthosis score of the observation group after surgery was significantly lower than that of the comparison group, indicating that unicondylar knee prosthesis replacement for knee osteoarthritis significantly improved knee flexion angle and tibial angle orthosis. This may be related to the onset of knee osteoarthritis often accompanied by intertrochanteric involvement, characterized by relatively mild involvement of the remaining femoral trochanteric compartments. The previously used tibial high osteotomy has a relatively small range of adaptation and can only play a role in correcting the force lines of the lower limb, so it is difficult to reduce the symptoms and cannot improve the functional situation of the knee joint [16]. It can effectively relieve the pain of the patient's knee and improve the knee flexion angle and their knee joint function [17]. The following points should be noted when performing unicondylar replacement: the key to force line reconstruction and inversion deformity correction lies in the proper selection of the prosthesis, minimizing the amount of osteotomy for the tibia during surgery, exposing only the diseased compartment without cutting the quadriceps muscle, avoiding damage to the knee extension function, facilitating postoperative rehabilitation, reducing adverse reactions, accurately placing the prosthesis, avoiding collision of the ligament and prosthesis, and removing the excess. Bone cement can be completely removed to reduce the occurrence of complications [18].

The VAS score in the observation group after surgery in our study was lower than that in the comparison group. However, the Lysholm score in the observation group after surgery was higher than that in the control group, indicating that unicondylar knee prosthesis replacement for osteoarthritis of the knee can improve the knee joint function in patients. When performing unicondylar replacement, it is important to note that the key to force line reconstruction and inversion deformity correction lies in properly selecting the prosthesis and minimizing the amount of osteotomy to the tibia during surgery. Exposing only the diseased compartment without cutting the quadriceps muscle also avoids damage to the knee extension function, facilitates postoperative rehabilitation, and reduces adverse effects [19]. It allows accurate prosthesis placement, avoiding collision of ligaments and prosthesis; it allows complete removal of excess bone cement, reducing complications [20]. The unicondylar knee prosthesis replaces only the medial compartment of the knee joint without damaging the lateral compartment and without affecting the normal knee structure. The knee proprioception is avoided and the cruciate ligament is preserved [21]. The amount of osteotomy is less compared to UKA, preserving an adequate amount of bone tissue, which is conducive to revision in patients in the distant future. The operation has the advantages of less intraoperative and postoperative bleeding, shorter hospital stay, and faster postoperative recovery [22]. The early follow-up study of patients with unicondylar knee prosthesis surgery proved that unicondylar knee prosthesis surgery has the advantages of less surgical injury, shorter operative time, less bleeding, and early weight-bearing activities [8]. The HSS scores, VAS scores, and knee range of motion (ROM) of the two groups of patients in this study at 7 days and 6 months after surgery showed that single condyle knee prosthesis replacement therapy for knee osteoarthritis recovered well. The HSS score is the more commonly used knee scoring method, and the HSS score increased significantly in both groups before and after surgery, indicating that both surgical methods were effective in treating unicompartmental osteoarthritis of the knee, achieving relatively satisfactory results and comparable efficacy in reducing pain levels in patients [23].

When we compared the complications of the two groups of patients in our study, the complication rate of patients in the observation group was significantly lower than that of the comparison group, indicating that patients with osteoarthritis of the knee treated with unicondylar knee prosthesis replacement had fewer complications. Lower extremity deep vein thrombosis is theoretically a serious complication common to both total knee replacement and unicondylar knee replacement, and dislodgment of lower extremity deep vein thrombosis such as embolization of the pulmonary artery is often life-threatening to patients and a common cause of death after arthroplasty [24]. In contrast, unicondylar knee replacements actually have a much lower incidence of lower extremity DVT and pulmonary embolism than total knee replacements due to their less invasive procedure and the advantage of early mobilization [25]. Common factors for lower extremity DVT include underlying patient disease, including the patient's own risk factors for lower extremity vascular disease, diabetic hypertension, dyslipidemia, long-term smoking, and heart valve disease [26].

Therefore, correct preoperative assessment and adequate preoperative preparation are beneficial to predict and prevent the formation of lower extremity deep venous thrombosis. Lack of correct and regular anticoagulation therapy before and after surgery will prolong the immobilization time of patients in bed. The need to actively encourage patients to move the affected limb actively in bed and get out of bed early after the drainage tube is removed after surgery are beneficial to prevent the formation of lower extremity deep vein thrombosis [27]. There are many risk factors for unicondylar knee replacement infection, usually the patient's own reasons such as the patient's recent history of intra-articular injections and punctures, the presence of diabetes, long-term hormone use or the presence of destructive autoimmune diseases, and septic infections in other parts of the body such as teeth and skin [7]. Intraoperative surgery that violates the principle of sterility can lead to bacterial invasion. Perioperative soft injuries affect local blood supply, bacterial colonization, and prolonged incision exposure [28]. Therefore, correct patient selection, preoperative education, and treatment of the primary disease are particularly important for the prevention of unicondylar knee replacement infection, followed by strict intraoperative aseptic operation, as little damage as possible to the surrounding soft tissues, and reasonable application of intraoperative and postoperative antibiotics are also effective methods of infection prevention [29]. Postoperative prosthesis loosening is a common cause of early failure of unicondylar knee replacement surgery, and knee unicondylar replacement prosthesis loosening is generally more common with tibial prosthesis [30].

The loosening of the prosthesis is mainly related to the surgical operation. Common intraoperative osteotomy is inaccurate, especially the tibial condyles are not ground thoroughly enough to leave a smooth cartilage surface, which can easily affect the adhesion of bone cement leading to postoperative femoral prosthesis loosening. Single-column prostheses are more prone to postoperative prosthesis loosening than double-column prostheses [16]. Secondly, too small selection of tibial prosthesis can also lead to loosening of the subprosthesis, etc. Increased tension in the lateral compartment due to overorthosis causing contralateral compartment osteoarthritis is also a common cause of failed revision of unicondylar knee replacements [31]. Studies have shown that by overorthosis of 5°, there is a corresponding 50% increase in the contralateral normal interventricular load, with a failure rate six times higher than in other cases [14]. Common reasons for this are as follows: preoperative patient selection and assessment is particularly important, primarily to determine the presence or absence of medial collateral ligament contracture by assessing the tension of the medial collateral ligament through stress tests and stress bitographs and secondarily to determine the integrity of the cartilaginous surface of the lateral interspace through stress bitographs [32]. Contracture of the medial collateral ligament and defective cartilage surfaces of the lateral interspace will cause early postoperative osteoarthritis of the lateral interspace, and intraoperative overcorrection, adjustment of gap balance by increasing the thickness of the movable spacer, and increasing the thickness of the movable spacer to prevent dislocation will lead to postoperative osteoarthritis of the lateral interspace due to increased tension of the lateral interspace [33]. Common causes of joint dislocation include key flexion-extension gap imbalance, mainly flexion-extension gap laxity, which is mostly seen in excessive periarticular soft tissue release, especially excessive medial collateral ligament release [19]. Bone cement and bone impingement is related to uncleared bone cement and bone flab in the posterior aspect of the joint, etc; inappropriate prosthesis selection, too small or too large prosthesis selection, and abnormal meniscus trajectory can lead to active meniscus dislocation [22].

There are some limitations in this study. First, the samples selected were all from patients treated or physically examined in our hospital, leading to a subjectivity in both inclusion and exclusion. There may be regional differences in the study results. Second, the small number of patients selected in this study may easily lead to biased results. Finally, it was impossible to study in-depth and follow up for a long time to understand the postoperative rehabilitation of patients with unicondylar osteoarthritis.

In conclusion, the clinical efficacy of unicondylar knee prosthesis replacement for knee osteoarthritis is better than that of unicondylar knee arthroplasty (UKA) treatment, and unicondylar knee prosthesis replacement can improve patients' knee function, significantly improve knee flexion angle, tibial angle orthosis, and joint mobility, and provide better postoperative recovery.

## Figures and Tables

**Figure 1:** AKS score, knee flexion angle, and tibial angle correction. All AKS score, knee flexion angle, and tibial angle correction data in this study were entered into excel software by the first author and the corresponding author, respectively, and independent sample *t*-test was performed with mean ± standard deviation. The results showed that the AKS score (a) and knee flexion angle (b) were higher in the observation group than in the comparison group after surgery; however, the tibial angle correction (c) was significantly lower in the observation group than in the comparison group after surgery, and this difference was statistically significant (*P* < 0.05).

**Figure 2:** Comparison of joint mobility. All the comparison of joint mobility data in this study were entered into excel software by the first author and the corresponding author, respectively, expressed as mean ± standard deviation, and an independent sample *t*-test was performed. The results showed that in the postoperative observation group, the VAS score (a) was lower than that of the control group, but the Lysholm score (b) of the observation group after surgery was higher than that of the control group, and the difference was statistically significant (*P* < 0.05).

**Figure 3:** Postoperative recovery comparison. All postoperative recovery comparison data in this study were entered into excel software by the first author and the corresponding author, respectively, expressed as mean ± standard deviation, and an independent sample *t*-test was performed. The results showed that in the two groups, the HSS score (a) and knee joint range of motion (ROM) (b) were statistically significant at 7 days and 6 months after surgery (*P* < 0.05).

**Figure 4:** Complications. All complication data in this study were entered into excel software by the first author and the corresponding author, respectively, represented by integers, and subjected to chi-square test. The results showed that the incidence of complications in the observation group was significantly lower than that in the control group. The difference was statistically significant (*P* < 0.05).

**Table 1:** Comparison of general data of the two groups of patients (*n*, ($\bar{x}\pm s$)).

Group	Gender (male/female)	Average age (years)	Body mass index (kg/m^2^)	Ahlback		
				I	II	III
Comparison group (50)	33/17	76.63 ± 10.32	28.31 ± 0.67	25	13	12
Observation group (50)	32/18	75.62 ± 10.31	28.33 ± 0.25	22	15	13
*χ* ^2^ */t*	0.044	0.490	-0.198	0.361	0.198	0.053
*P*	0.834	0.625	0.844	0.548	0.656	0.817

## Data Availability

The datasets used and analyzed during the current study are available from the corresponding author upon reasonable request.
